# Urinary PCA3 a Superior Diagnostic Biomarker for Prostate Cancer among Ghanaian Men

**DOI:** 10.1155/2022/1686991

**Published:** 2022-10-07

**Authors:** Bismark Opoku Mensah, Linda Ahenkorah Fondjo, W. K. B. A. Owiredu, Ben Adusei

**Affiliations:** ^1^Department of Molecular Medicine, KSMD, KNUST, Ghana; ^2^Urology Unit, 37 Military Hospital, Accra, Ghana

## Abstract

**Introduction:**

Prostate cancer is one of the most commonly diagnosed cancers in men. Prostate-specific antigen (PSA) has been the biomarker of choice for screening and diagnosis of prostate cancer. However, inefficiencies exist with its diagnostic capabilities. This study thus evaluated the diagnostic and prognostic potential of urinary PCA3 as an alternative biomarker for prostate cancer in the Ghanaian population.

**Methods:**

A hospital-based cross-sectional study was conducted at the Urology Department of the 37 Military Hospital, Accra, Ghana. A total of 237 participants aged 40 years and above with any form of suspected prostate disorder were recruited into the study after written informed consent was obtained. Total serum PSA levels was measured using the electrochemiluminescence method and transrectal ultrasound-guided systematic core needle biopsies were obtained from each study participant. Receiver operating characteristic curve (ROC) analysis was used to evaluate the diagnostic accuracies of serum PSA, DRE, and PCA3 as diagnostic tools for prostate cancer. These three diagnostic tools were also evaluated in various combinations to ascertain the combinations with the best diagnostic accuracy.

**Results:**

Prostate cancer was diagnosed in 26.6% of the participants. Benign prostate hyperplasia and prostatitis were diagnosed in 48.5% and 24.9% participants, respectively. DRE had a sensitivity of 93.7% and a specificity of 12.1%. PSA had a sensitivity of 92.1% and a specificity of 16.1%. PCA3 had a sensitivity of 57.1% and a specificity of 85.6% and showed a better accuracy (AUC = 83.0) compared to PSA (AUC = 60.0) and DRE (AUC = 65.0) as individual diagnostic tools. The combination of DRE+PCA3 score had the best diagnostic accuracy (AUC = 0.80) with a sensitivity and specificity of 60.3% and 80.5%, respectively.

**Conclusion:**

The urinary PCA3 assay showed a better diagnostic performance compared to serum PSA and DRE. PCA3 as a stand-alone and in combination with DRE could be a suitable complimentary marker in diagnosis and management of prostate cancer.

## 1. Introduction

Prostatic carcinoma is one of the cancers mostly diagnosed in men and a leading cause of cancer death in men. It is estimated that there are over seventy-five million prevalent cases, twenty-seven million incident cases, and seventeen million deaths expected globally by 2030 [1–3]. Across the African continent, countries such as Uganda, South Africa, Nigeria, Ghana, and Zimbabwe, the incidence of prostate cancer is reported to increase among men between the ages of 40 and 70 years [4, 5].

In Ghana, the clinical and laboratory screening for prostate cancer is mostly done with prostate-specific antigen (PSA) and digital rectal examination (DRE). Screening for prostate cancer with PSA has largely led to a decrease in prostate cancer mortality [6] and assisted clinicians in case management of men with prostate cancer worldwide. However, some inefficiencies have been reported with the use of PSA for prostate cancer screening and diagnosis. PSA is known to be elevated in prostatitis, trauma, benign prostatic hyperplasia, and other pathological and physiological conditions of the urinary system [7]. This makes the continuous reliance on PSA for clinical decision making in prostate cancer cases problematic particularly in the Ghanaian population where it is still the main diagnostic criteria. Considering the heterogenicity of prostate carcinoma and the factors that influence the release of PSA from the prostate and the limitations that exist with the use of PSA, it is imperative that the introduction of other biomarkers with higher sensitivity and specificity is explored to minimize overdiagnosis associated with PSA screening. One of such molecular biomarkers that has shown significant prospects in improving on some of the limitations of PSA is prostate cancer gene 3 (PCA3) [8, 9].

Prostate cancer gene 3 (PCA3) is specific to the prostate gland and expressed significantly in cancerous prostate tissues compared to benign prostate tissues [10]. This may give PCA3 a cancer specificity that may be lacking with PSA. PCA3 levels in the urine is associated with the extent of metastatic activity of cancerous cells in the prostate, which suggests that PCA3 could be valuable in the diagnosis of prostatic carcinomas [11].

The clinical use of PCA3 urine assay as a diagnostic and screening tool for prostate cancer in European and US men is well documented [12]. However, scanty or no clinical data is currently available on the potential of the prostate cancer gene 3 (PCA3) urine assay as a screening and/or diagnostic tool in other population especially in the African population where the incidence of prostate cancer is on the rise. This study evaluated the potential of PCA3 as a diagnostic biomarker and compared the performance characteristics of urine PCA3 and serum PSA as diagnostic tools for prostate carcinomas in Ghanaian men.

## 2. Methods

### 2.1. Study Design and Setting

This study was a hospital-based cross-sectional study conducted at the Urology Department of the 37 Military Hospital, Accra, Ghana, from February 2019 to August 2020. The 37 Military Hospital is a teaching hospital located in Accra, the capital city of Ghana, and has several departments including Surgical, Medical, Paediatrics, Obstetrics, Gynecology, Dental, Pathology, Pharmacy, Physiotherapy, and Urology.

### 2.2. Study Population and Participants Selection

The study employed a nonprobability convenience sampling technique to recruit 237 men who visited the Urology Unit of the 37 Military Hospital. Men forty years and above reporting to the Urology Department for the first time with any form of suspected prostate disorder were eligible for the study. Men who had elevated total serum PSA (≥4.0 ng/ml) and or abnormal results on DRE were recruited as study participants after giving written informed consent. Excluded participants were men below 40 years of age and men who were taking drugs for the treatment or management of any urologic disorder.

### 2.3. Ethical Considerations

Ethical approval for the study was obtained from the Committee on Human Research, Publication, and Ethics of the School of Medicine and Dentistry (SMD), Kwame Nkrumah University of Science and Technology (KNUST) (CHRPE/AP/537/19), and the ethical review board of the 37 Military Hospital (37MH-IRB IPN/306/2019), respectively. Participants enrolled onto the study willingly after written informed consent. All experiments were conducted in accordance with the Declaration of Helsinki (1964).

### 2.4. Questionnaire Administration

A well-structured and validated questionnaire was designed and administered to each study participant to obtain sociodemographic information including age, occupation, educational status, ethnicity, and behavioural activities (smoking and alcohol consumption). Smoking was defined as smoking at least one cigarette a day and alcohol consumption was defined as drinking at least a bottle of any alcoholic liquor weekly.

The medical history of each participant was taken. These included a history of other chronic illnesses such as diabetes, hypertension, kidney disease, duration of such illness, medications, family history of chronic diseases, and a history of present and past medication. This information was verified from the medical records of each participant.

### 2.5. Blood Sample Collection

About five (5) ml of blood was drawn from the antecubital vein of participants observing all aseptic protocols prior to DRE and ultrasound scan examinations. The blood sample was dispensed into a plain-gel tube and then centrifuged, and the sera obtained were stored at -80°C and used for measurement of PSA levels.

### 2.6. PSA Assay

Total PSA was measured using the electrochemiluminescence method (Cobas e411 Analyzer, Roche Diagnostics, Germany). The Cobas e411 automates the immunoassay reactions using a sandwich electrochemiluminescent immunoassay standardized using the Reference Standard/WHO 96/670.

### 2.7. Digital Rectal Examination (DRE)

Digital rectal examination was carried out on all participants by a certified urologist. The DRE was performed to evaluate prostate shape, size, consistency, presence or absence of nodules, symmetry, edge, tenderness, or the presence of any rectal mass.

### 2.8. Ultrasound Scan Imaging

Transrectal ultrasonography (TRUS) was performed on all study participants by a certified sonographer using the Mindray DP-50 digital ultrasound scan machine (Shenzhen Mindray Bio-Medical Electronics, China) with probes of frequency 5-12 MHz to determine the volume and the configuration of the prostate.

### 2.9. Prostate Cancer Antigen 3 (PCA3) Urine Assay

About 5 ml of first-catch urine samples was collected immediately after DRE had been performed on each study participant. The PCA3 assay kit (Gen-Probe Inc., San Diego, CA, USA) was used to measure the mRNA concentrations in the urine samples, and a PCA3 score based on the ratio of urine PCA3 to PSA mRNA was determined.

### 2.10. Prostate Biopsy

Transrectal ultrasound-guided systematic core needle prostate biopsies were taken from study participants who had PSA ≥ 4.0 ng/ml or abnormal and or suspicious results on DRE. The prostate biopsies were stained and examined by a certified pathologist who had no prior knowledge of the clinical conditions of the participants.

### 2.11. Statistical Analysis

Statistical analyses were performed using SPSS ver. 22.0 (IBM, Armonk, NY, USA). Descriptive statistics were performed for demographic variables and were expressed as mean ± standard deviation (SD) for continuous variables with normal distribution. In cases of asymmetrical distribution, median and interquartile (IQR) values were used. Variables such as age, PSA, and prostate volume were compared using chi (*χ*^2^) tests, *t*-test, and Mann–Whitney *u*-test. Nonparametric values were compared using the Fisher exact test. ROC analysis was used to evaluate the accuracies in predicting positive outcomes and performance of combination of the tests. Multivariate logistic regression analyses were used to evaluate the relationships between PCA3 score, Gleason score, and percentage positive biopsy cores; a *p* value ≤ 0.05 was considered significant.

## 3. Results

Prostate cancer was detected in 63 (26.6%) out of the 237 participants. Benign prostatic hyperplasia and prostatitis were the major nonmalignant conditions diagnosed in a greater number of the participants. Prostatitis and benign prostatic hyperplasia were diagnosed in 59 (24.9%) and 115 (48.5%) participants, respectively. Benign prostatic hyperplasia (37.4%) and prostatitis (44.1%) were diagnosed predominantly among participants within age group 50–59 years. Prostate cancer (34.9%) was most predominant among participants within the age group 70–79 years (Table 1).

A higher proportion, 96 (55.2%) participants without prostate cancer and 27 (42.9%) cancer subjects were within the PSA range 4.0-10.0 ng/ml. Majority of the participants with prostate cancer had increased PSA levels (>20 ng/ml) compared to their counterparts without prostate cancer (Table 2). As expected, there was a significant difference in total serum PSA (*p* = 0.025) between participants with and without prostate cancer. A greater proportion (71.8%) of participants without prostate cancer had a PCA3 score < 15.0. Participants with prostate cancer had increased PCA3 score from 15.0 to 60.0 with majority (28.6%) of them having a PCA3 score greater than 60.0 (Table 2). Digital rectal examination detected 50 (21.1%) positive and 187 (78.9%) negative participants. There was a significant difference in PCA3 scores and DRE findings between subjects with and without prostate cancer (*p* = 0.0001) There was no significant difference in prostate volume (*p* = 0.210) between subjects with and without prostate cancer.

Serum PSA had a sensitivity of 92.1% and a specificity of 16.1% at a PSA cut-off value of 4.0 ng/ml with positive and negative predictive values of 28.4% and 84.8%, respectively. Using a PCA3 score cut-off value of 30.0, PCA3 score had a sensitivity of 57.1% and a specificity of 85.6% with a negative predictive value of 84.7%. DRE had a sensitivity and specificity of 66.7% and 60.3%, respectively, and a negative predictive value of 83.6% (Table 3). ROC curve analysis performed on the performance of PSA, PCA3 score, and DRE as diagnostic methods with biopsy as the reference method (Figure 1) gave an area under the curve (AUC) of 0.60, 0.83, and 0.65, respectively. Among the three prostate cancer diagnostic tests, PCA3 score performed better yielding an AUC of 0.83 (95% CI: 0.74 to 0.90) (Figure 1).

Multivariate logistic regression analysis showed that high PCA3 score (OR: 1.621, *p* = 0.001) and high levels of serum PSA (OR: 1.110, *p* = 0.031) had a significant correlation with high Gleason score (Table 4). An increase in the PCA3 score was found to be associated and positively correlated (*r* = 1.169) with an increase in prostate cancer incidence (*p* < 0.0001) (Figure 2).

PCA3 cut-off score of 10 had the highest sensitivity (93.7%) with a specificity of 48.9%, and a cut-off of 50 had the lowest sensitivity (39.7%) and highest specificity (100.0%). The sensitivity and specificity were 69.8% and 72.4%, respectively, at a cut-off of 20. A cut-off of 30 combined the greatest cancer sensitivity (57.1%) and specificity (85.6%) (diagnostic accuracy = 0.78 and Youden index of 0.53). PCA3 cut-off score of 40 yielded a sensitivity of 44.4% and a specificity of 96.0%. Diagnostic sensitivity decreased with increasing PCA3 score as with negative predictive values while specificity and positive predictive values generally increased with increasing PCA3 scores (Table 5).

The combination of PSA and DRE (PSA+DRE) had a sensitivity of 100% and a specificity of 2.9%. PSA+PCA3 score combination had a sensitivity and specificity of 71.4% and 52.9%, respectively. The combination of DRE and PCA3 score (DRE+PCA3 score) had a sensitivity of 60.3% and a specificity of 80.5%. The three combined parameters (PSA+DRE+PCA3 score) had a sensitivity and specificity of 60.3% and 78.2%, respectively (Table 6). The combination of DRE+PCA3 score had the best diagnostic accuracy (*AUC* = 0.80) (Figure 3) with a sensitivity and specificity of 60.3% and 80.5%, respectively (Table 6).

## 4. Discussion

In the Ghanaian population, prostate-specific antigen (PSA) and digital rectal examination (DRE) are the key screening and diagnostic protocols for making clinical decisions when prostate cancer is suspected in men. The use of PSA and DRE as the basis for recommending patients for biopsy often leads to patients being subjected to unnecessary biopsies due to the lack of specificity of PSA and DRE. Thus, we evaluated the diagnostic and prognostic potential of urinary prostate cancer gene 3 (PCA3) as a biomarker for diagnosing prostate cancer and compared the performance characteristics of serum PSA and urinary prostate cancer gene 3 (PCA3). Prostate-specific antigen (PSA), digital rectal examination (DRE), and urinary prostate cancer gene 3 (PCA3) score were used as the diagnostic tools with biopsy as the reference diagnostic tool in the assessment of prostate disorders in the participants.

In this study, 26.6% presented with prostate cancer among the study participants, a finding consistent with the study by Yeboah et al. in Kumasi, Ghana. A systematic review and a meta-analysis of forty (40) studies spreading across 16 African countries also reported a pooled prevalence of prostate cancer consistent with our findings [1]. However, reports from a population-based study from the Kumasi Cancer Registry (KsCR) [13] and a population-based study among West Africans [14] reported a much lower prostate cancer incidence of 13.2% and 7.0%, respectively. A small proportion, representing 6.4% of the participants between the ages 40 and 49 years were diagnosed with prostate cancer in this current study; this is in agreement with the assertion that only about 1 out of 350 men under the age of 50 years is likely to be diagnosed with prostate cancer [15]. Furthermore, this finding is also consistent with the SEER Cancer Statistics Review in 2013 which reported a lower incidence of prostate carcinoma among men between ages 40 and 49 years [16].

Majority, 42.9%, of the men diagnosed with prostate cancer were within the PSA range 4.0 ng/ml to 10.0 ng/ml. This is in conformity with prospective cohort studies in the United States and China by Jue et al. and Tang et al., respectively, who reported that about 44% of prostate cancer patients had PSA values ranged between 4.0 and 10.0 ng/ml [17, 18]. Moreover, a higher proportion of men diagnosed with nonmalignant conditions of the prostate (BPH and prostatitis) were also within the PSA range 4.0 ng/ml to 10.0 ng/ml (Table 2). This supports the fact that many nonmalignant pathologies other than prostate cancer lead to increase in total serum PSA [19–21]. In this current study, the sensitivity and specificity of PSA for prostate cancer detection were 92.1% and 16.1%, respectively, at a PSA cut-off of 4.0 ng/ml (Table 3). This agrees with findings of several studies across the globe which report very high sensitivity with low specificity for PSA in the detection of prostate cancers [22–24].

Our study found that the PCA3 scores for men diagnosed with prostate cancer were significantly higher than those for those diagnosed with nonmalignant conditions of the prostate. To predict the accuracy for predicting the accuracy for detecting prostate cancer, we report that PCA3 had an AUC of 83.0 compared to 59.5 for serum PSA (Figure 1), with urine PCA3 showing significant association with prostate cancer detection. Our findings are consistent with findings by Auprich et al. and Ploussard et al., who observed that PCA3 is valuable in detecting prostate cancer in men scheduled for initial biopsies [25, 26].

Chronic inflammation is a known risk factor for several forms of human cancer and now regarded as an “enabling characteristic” of human cancer [27, 28]. Considering the heterogeneous nature of bacterial and nonbacterial prostate inflammation and the recurrence rates [29], chronic inflammation of the prostate may have an effect on the diagnostic accuracy of urinary PCA3 and may impact the accuracy of urinary PCA3 in predicting prostate cancer. However, in this current study, the effect of chronic inflammation on the accuracy of urinary PCA3 was not explored.

In this current study, urinary PCA3 had similar negative predictive value (NPV) of 84.7% compared with PSA (84.8%) and DRE (84.0%) but significantly higher positive predictive value (PPV) of 59.0% corroborating the findings of three community-based studies on men undergoing initial and repeated prostate biopsies [30–32]. PCA3 score also correlated significantly with the probability to detect a positive biopsy (Figure 2) supporting the hypothesis that the probability of detecting prostate cancer increases with increasing PCA3 scores [8, 33]. However, a multiparametric MRI was not used in the detection of prostate cancer in this study and thus acknowledged as a limitation of the study. Multiparametric magnetic resonance imaging (mpMRI) with or without targeted biopsy has a well-established role in the detection of clinically significant PCa (csPCa) and an appealing alternative to transrectal ultrasonography (TRUS) biopsy [34–36] that was employed in this current study. Compared with systematic transrectal ultrasonography-guided biopsy, mpMRI is associated with a 57.0% improvement in the detection of clinically significant PCa and a 77% reduction in the number of cores taken per procedure [35, 37]. Alkasab et al. in evaluating the performance of PCA3 and MpMRI also reported an NPV of 40% and 83%, respectively. However, adding mpMRI to high PCA3 scores augmented the NPV to 95% [38]. In comparing mpMRI, SelectMDx, and PSA as separate tools and in various combinations, the association of mpMRI and SelectMDx was reported to have the best performance in predicting PCa and csPCa after biopsy [39]. Thus, an MRI first pathway may have influenced the performance and accuracy of urinary PCA3 in the detection of prostate cancer in the Ghanaian population.

Our findings suggest that PCA3 may not be a complete replacement for PSA as the appropriate choice of test for prostate cancer especially in the Ghanaian population but may however serve as a complimentary diagnostic biomarker which would be very beneficial in the management and treatment of malignant and nonmalignant prostate conditions.

There are contrasting reports and differing views regarding the optimal cut-off of PCA3 values for discriminating men having prostate cancer and those with benign prostate conditions [40]. The PCA3 assay used in this study proposes a cut-off of 35 as the optimal threshold for improved sensitivity and specificity [41]. However, several experimental studies have suggested that the optimal threshold of PCA3 may be dependent on population characteristics [42–45]. In this current study, a PCA3 score of 30.0 gave the best combination of sensitivity and specificity among Ghanaian men (Table 5). Merola et al. and Luo et al. documented a much lower cut-off of 20.0 among Italian and Chinese men [41, 46], while multicentered hospital-based studies in Europe by Marks et al. and Roobol et al. reported specificities above 90.0% at a cut-off of 100.0 [30, 47].

In this study, high levels of serum PSA and increased PCA3 score significantly correlated with Gleason score; while age and prostate volume showed no significant correlation with Gleason score (Table 4). This is in consonance with reports on men with suspected prostatic carcinoma in the Zhejiang province of China [48]. This finding also supports the opinion expressed by Groskopf et al., that PCA3 as a tissue-based overexpressed biomarker can be a promising urinary marker that can support the diagnosis and management of prostate cancer in clinical practice [49]. Additionally, this study supports the report by De Luca and colleagues which suggested that PCA3 could be a main determinant for prostatitis, high-grade prostatic intraepithelial neoplasia (HG-PIN), and prostate cancer [50]. Several studies have reported that patients with small foci of prostate cancer mostly benefit from active surveillance than from immediate treatment. It has been suggested that patients with small foci of prostate cancers should be placed on active surveillance than on chemotherapy [51, 52]. However, the major concerns of most clinicians in placing patients under active surveillance are the uncertainty in the use of PSA and or DRE as the basis for such decisions [53]. From the findings of this study, we suggest that PCA3 holds the potential valuable in deciding which patients will benefit from active surveillance or immediate treatment.

Often in clinical settings, a single biomarker is not sufficient to accurately assess the clinical significance of prostate cancer at the time of diagnosis. This is due to the heterogeneity in the pathogenesis of prostate cancer [54], a fact that has informed the opinion that the combination of multiple markers and diagnostic protocols could improve the rates of detection of prostatic carcinomas [54, 55]. In assessing the performance of combined diagnostic tools in detecting prostate cancer, results from this study show that combinations of diagnostic tests improve the rates of detection of prostate cancers compared to the use of single diagnostic tests (Table 6), corroborating the findings by Descotes and Dimakakos et al. [54, 55]. Another descriptive retrospective studies also reported similar findings among Algerian men [56]. Shimizu et al. also observed a higher detection rate for prostate cancer using a combination of PSA and DRE as compared to when DRE and PSA were used as single diagnostic tools [57].

Positive predictive value is a parameter that is very essential in the assessment of cancer detection as it gives vital clinical information on the frequency of redundant biopsies [58–60]. In this study, DRE+PCA3 combination had the highest positive predictive value followed by PSA+DRE+PCA3 combinations (Table 6). These findings suggest that the addition of urinary PCA3 to the current routine diagnostic protocols in Ghana can improve the outcome of prostate cancer screening and reduce the number of patients who may have to go through unnecessary invasive biopsy procedures.

## 5. Conclusion

The urinary PCA3 assay showed a better diagnostic performance compared to serum PSA and DRE. Urinary PCA3 assay can facilitate the selection of high-risk men who may benefit from prostate biopsy. PCA3 urine assay could therefore be a useful marker in detecting prostate cancer in our population.

## Figures and Tables

**Figure 1:** Receiver operating characteristic (ROC) curve analysis for the diagnostic performance of serum PSA, PCA3 score, and DRE.

**Figure 2:** Biopsy outcome with PCA3 score.

**Figure 3:** Receiver operating characteristic (ROC) curve analyses showing the accuracy of the various combinations of the diagnostic tools.

**Table 1:** Distribution of prostate disorders among the study participants.

Variable	Biopsy results			
Age groups (years)	PCa *n* (%)	BPH *n* (%)	Prostatitis *n* (%)	Number (*n*)
40–49	4 (6.4%)	12 (10.4%)	7 (11.9%)	23
50–9	13 (20.6%)	43 (37.4%)	26 (44.1%)	82
60–69	17 (27.0%)	34 (29.6%)	17 (28.8%)	68
70–79	22 (34.9%)	22 (19.1%)	8 (15.5%)	52
>80	7 (11.1%)	4 (3.5%)	1 (1.7%)	12
Total	63	115	59	237

PCa: prostate cancer; BPH: benign prostatic hyperplasia.

**Table 2:** Comparison of diagnostic parameters among the study participants.

Variables	PCa (*n* = 63)	Without PCa (*n* = 174)	*p* value
PSA (ng/ml) (median, IQR)	12.1 (6.7–24.2)	8.7 (6.2–14.5)	0.025
PSA category (ng/ml)			
4-10	27 (42.9%)	96 (55.2%)	0.0001
10.1-20	16 (25.4%)	60 (34.5%)	
>20	20 (31.7%)	18 (10.3%)	
PCA3 score (median, IQR)	42.8 (19.9–64.8)	10.1 (6.3–16.7)	0.0001
<15	7 (11.1%)	125 (71.8%)	0.0001
15.1-30.0	14 (22.2%)	37 (21.3%)	
30.1-45.0	11 (17.5%)	12 (6.9%)	
45.1-60.0	13 (20.6%)	0	
>60.0	18 (28.6%)	0	
DRE findings			
Positive	27 (42.9%)	23 (13.2%)	0.0001
Negative	36 (57.1%)	151 (86.8%)	
Prostate volume (ml) (median, IQR)	35.1 (29.8–45.9)	33.9 (28.8–40.1)	0.210
Prostate volume category (ml)			
≤40	39 (61.90%)	128 (73.60%)	0.230
40-80	20 (31.70%)	38 (21.80%)	
>80	4 (6.30%)	8 (4.60%)	

PSA: prostate-specific antigen; PCA3: prostate cancer antigen 3; DRE: digital rectal examination; IQR: interquartile range.

**Table 3:** Diagnostic performance of total serum PSA, PCA3 score, and DRE.

Variable	Sensitivity (95% CI)	Specificity (95% CI)	PPV (%)	NPV (%)	TP	TN	FP	FN
PSA (ng/ml)	92.1 (82.2–96.9)	16.1 (11.4–22.4)	28.4	84.8	58	28	146	5
PCA3 score	57.1 (44.9–68.6)	85.6 (79.6–90.1)	59.0	84.7	36	149	25	27
DRE	93.7 (84.2–97.9)	12.1 (8.0–17.8)	27.7	84.0	59	21	153	4

PSA: prostate-specific antigen; PCA3: prostate cancer antigen 3; DRE: digital rectal examination; CI: confidence interval; PPV: positive predictive value; NPV: negative predictive value; TP: true positive; TN: true negative; FP: false positive; FN: false negative.

**Table 4:** Association between age, PCA3 score, serum PSA, prostate volume, and Gleason score of participants with prostate cancer.

Gleason score					
Variable	≤7.0 (*n* = 38)	≥8.0 (*n* = 25)	OR	95% CI	*p* value
Age (years)	65.4 ± 10.8	67.8 ± 8.9	0.042	63.6–68.9	0.14
PCA3 score (median, IQR)	31.1 (15.9-46.4)	67.8 (49.5-80.4)	1.621	38.2-50.5	0.001
PSA (median, IQR)	8.5 (5.6-27.8)	12.9 (7.8-24.1)	1.110	14.3-25.1	0.031
Prostate volume (ml) (median, IQR)	35.4 (31.5-44.0)	32.1 (27.4-46.8)	0.962	35.8-43.6	0.82

SD: standard deviation; OR: odds ratio; IQR: interquartile ratio; CI: confidence interval.

**Table 5:** PCA3 score sensitivity and specificity at various cut-off points.

PCA3 score cut-off	Sensitivity (%)	Specificity (%)	PPV (%)	NPV (%)	AUC (95% CI)
10	93.7	48.9	39.9	95.5	0.570 (0.49–0.65)
20	69.8	72.4	47.8	86.9	0.713 (0.65–0.78)
30	57.1	85.6	59.0	84.7	0.830 (0.74–0.90)
40	44.4	96.0	80.0	82.7	0.70 (0.62–0.75)
50	39.7	100.0	100	82.1	0.708 (0.63–0.79)

AUC: area under the curve; CI: confidence interval; PPV: positive predictive value; NPV: negative predictive value.

**Table 6:** Diagnostic performance of combination of diagnostic tools for prostate cancer.

Variable	Sensitivity (95% CI)	Specificity (95% CI)	PPV (%)	NPV (%)	TP	TN	FP	FN
PSA + DRE	100.0 (92.9-100)	2.9 (1.1–6.8)	27.2	100.0	63	5	169	0
PSA + PCA3 score	71.4 (59.2–81.1)	52.9 (45.5–60.1)	35.4	83.6	45	92	82	18
DRE+PCA3 score	60.3 (48.0–71.4)	80.5 (73.9–85.7)	52.8	84.8	38	140	34	25
PSA+DRE+PCA3 score	60.3 (48.0–71.4)	78.2 (71.4–83.7)	50.0	84.5	38	136	38	25

PSA: prostate-specific antigen; PCA3: prostate cancer antigen 3; DRE: digital rectal examination; CI: confidence interval; PPV: positive predictive value; NPV: negative predictive value; TP: true positive; TN: true negative; FP: false positive; FN: false negative.

## Data Availability

The datasets used and/or analyzed in this study are within the manuscript.

## References

[1] Adeloye D., David R. A., Aderemi A. V. (2016). An estimate of the incidence of prostate cancer in Africa: a systematic review and meta-analysis. *PLoS One*.

[2] Ferlay J., Shin H. R., Bray F., Forman D., Mathers C., Parkin D. M. (2010). Estimates of worldwide burden of cancer in 2008: GLOBOCAN 2008. *International Journal of Cancer*.

[3] Parkin D. M., Ferlay J., Hamdi-Cherif M. (2003). *Cancer in Africa. IARC Scientific Publication No. 153.*.

[4] Parkin D. M., Wabinga H., Nambooze S. (2001). Completeness in an African cancer registry. *Cancer Causes & Control*.

[5] Yeboah F., Acheampong E., Gyasi-Sarpong C. K. (2018). Nomogram for predicting the probability of the positive outcome of prostate biopsies among Ghanaian men. *African Journal of Urology*.

[6] Tabayoyong W., Abouassaly R. (2015). Prostate cancer screening and the associated controversy. *The Surgical Clinics of North America*.

[7] Barry M. J. (2001). Prostate-specific–antigen testing for early diagnosis of prostate cancer. *New England Journal of Medicine*.

[8] Prensner J. R., Rubin M. A., Wei J. T., Chinnaiyan A. M. (2012). Beyond PSA: the next generation of prostate cancer biomarkers. *Science Translational Medicine*.

[9] Saini S. (2016). PSA and beyond: alternative prostate cancer biomarkers. *Cellular Oncology*.

[10] Bussemakers M. J., van Bokhoven A., Verhaegh G. W. (1999). DD3: a new prostate-specific gene, highly overexpressed in prostate cancer. *Cancer Research*.

[11] Galasso F., Giannella R., Bruni P. (2010). PCA3: a new tool to diagnose prostate cancer (PCa) and a guidance in biopsy decisions. Preliminary report of the UrOP study. *Archivio Italiano di Urologia, Andrologia*.

[12] Adhyam M., Gupta A. K. (2012). A review on the clinical utility of PSA in cancer prostate. *Indian Journal of Surgical Oncology*.

[13] Laryea D. O., Awuah B., Amoako Y. A. (2014). Cancer incidence in Ghana, 2012: evidence from a population-based cancer registry. *BMC Cancer*.

[14] Hsing A. W., Yeboah E., Biritwum R. (2014). High prevalence of screen detected prostate cancer in West Africans: implications for racial disparity of prostate cancer. *The Journal of Urology*.

[15] Perdana N. R., Mochtar C. A., Umbas R., Hamid A. R. (2016). The risk factors of prostate cancer and its prevention: a literature review. *Acta Medica Indonesiana*.

[16] Howlader N. N., Noone A. M., Krapcho M. (2013). *SEER cancer statistics review, 1975–2010*.

[17] Jue J. S., Barboza M. P., Prakash N. S. (2017). Re-examining prostate-specific antigen (PSA) density: defining the optimal PSA range and patients for using PSA density to predict prostate cancer using extended template biopsy. *Urology*.

[18] Tang P., Du W., Xie K. (2013). Transition zone PSA density improves the prostate cancer detection rate both in PSA 4.0–10.0 and 10.1–20.0 ng/ml in Chinese men. *Urologic Oncology: Seminars and Original Investigations*.

[19] Bley D., Kaplan S., Johnson D. (1992). The strengths and limitations of PSA: where we stand. *Reliability Engineering & System Safety*.

[20] Jemal A., Siegel R., Ward E. (2008). Cancer statistics, 2008. *CA: a Cancer Journal for Clinicians*.

[21] Marks L. S., Bostwick D. G. (2008). Prostate cancer specificity of PCA3 gene testing: examples from clinical practice. *Reviews in Urology*.

[22] Lojanapiwat B., Anutrakulchai W., Chongruksut W., Udomphot C. (2014). Correlation and diagnostic performance of the prostate-specific antigen level with the diagnosis, aggressiveness, and bone metastasis of prostate cancer in clinical practice. *Prostate International*.

[23] Wadie B., Abdelfatah E. S. A., Emara S. E., Bazeed M. A. (2003). The discriminative ability of percent free PSA in patients with PSA> 10 ng/ml. *African Journal of Urology*.

[24] Yunusa B., Abdullahi M., Mashi S. A., Aji S. A., Alhassan S. U. (2017). Determination of the sensitivity and specificity of serum prostate-specific antigen in the diagnosis of prostrate cancer in Kano, Northwestern Nigeria. *Nigerian Journal of Basic and Clinical Sciences*.

[25] Auprich M., Chun F. K. H., Ward J. F. (2011). Critical assessment of preoperative urinary prostate cancer antigen 3 on the accuracy of prostate cancer staging. *European Urology*.

[26] Ploussard G., Durand X., Xylinas E. (2011). Prostate cancer antigen 3 score accurately predicts tumour volume and might help in selecting prostate cancer patients for active surveillance. *European Urology*.

[27] Roberts R. O., Bergstralh E. J., Bass S. E., Lieber M. M., Jacobsen S. J. (2004). Prostatitis as a risk factor for prostate cancer. *Epidemiology*.

[28] Sfanos K. S., De Marzo A. M. (2012). Prostate cancer and inflammation: the evidence. *Histopathology*.

[29] Busetto G. M., Giovannone R., Ferro M. (2014). Chronic bacterial prostatitis: efficacy of short-lasting antibiotic therapy with prulifloxacin (Unidrox®) in association with saw palmetto extract, lactobacillus sporogens and arbutin (Lactorepens®). *BMC Urology*.

[30] Marks L. S., Fradet Y., Lim Deras I. (2007). PCA3 molecular urine assay for prostate cancer in men undergoing repeat biopsy. *Urology*.

[31] Schilling D., Hennenlotter J., Munz M., Bökeler U., Sievert K. D., Stenzl A. (2010). Interpretation of the prostate cancer gene 3 in reference to the individual clinical background: implications for daily practice. *Urologia Internationalis*.

[32] Vlaeminck-Guillem V., Ruffion A., André J., Devonec M., Paparel P. (2010). Urinary prostate cancer 3 test: toward the age of reason?. *Urology*.

[33] Crawford E. D., Ventii K. H., Shore N. D. (2016). New markers for prostate cancer detection and prognosis. *Prostate Cancer*.

[34] Ghai S., Haider M. A. (2015). Multiparametric-MRI in diagnosis of prostate cancer. *Indian Journal of Urology*.

[35] Klotz L., Chin J., Black P. C. (2021). Comparison of multiparametric magnetic resonance imaging–targeted biopsy with systematic transrectal ultrasonography biopsy for biopsy-naive men at risk for prostate cancer: a phase 3 randomized clinical trial. *JAMA Oncology*.

[36] Penzkofer T., Tempany-Afdhal C. M. (2014). Prostate cancer detection and diagnosis: the role of MR and its comparison with other diagnostic modalities–a radiologist's perspective. *NMR in Biomedicine*.

[37] Saltman A., Zegar J., Haj-Hamed M., Verma S., Sidana A. (2021). Prostate cancer biomarkers and multiparametric MRI: is there a role for both in prostate cancer management?. *Therapeutic Advances in Urology*.

[38] Alkasab T., Ahmad A., Rechard P. (2016). MP53-12 the role of prostate cancer antigen 3 (PCA3) test and multi-parametric prostatic magnetic resonance imaging (MPMRI) among patients with prior negative biopsy: correlation with radical prostatectomy pathology. *The Journal of Urology*.

[39] Maggi M., del Giudice F., Falagario U. G. (2021). SelectMDx and multiparametric magnetic resonance imaging of the prostate for men undergoing primary prostate biopsy: a prospective assessment in a multi-institutional study. *Cancers*.

[40] Ramos C. G., Valdevenito R., IvonneVergarac P. A., Sanchez C., Fulla J. (2013). PCA3 sensitivity and specificity for prostate cancer detection in patients with abnormal PSA and/or suspicious digital rectal examination. First Latin American experience. *Urologic Oncology: Seminars and Original Investigations*.

[41] Merola R., Tomao L., Antenucci A. (2015). PCA3 in prostate cancer and tumor aggressiveness detection on 407 high-risk patients: a National Cancer Institute experience. *Journal of Experimental & Clinical Cancer Research*.

[42] Bollito E., de Luca S., Cicilano M. (2012). Prostate cancer gene 3 urine assay cutoff in diagnosis of prostate cancer: a validation study on an Italian patient population undergoing first and repeat biopsy. *Analytical and Quantitative Cytology and Histology*.

[43] Gittelman M. C., Hertzman B., Bailen J. (2013). PCA3 molecular urine test as a predictor of repeat prostate biopsy outcome in men with previous negative biopsies: a prospective multicenter clinical study. *The Journal of Urology*.

[44] Haese A., de la Taille A., van Poppel H. (2008). Clinical utility of the PCA3 urine assay in European men scheduled for repeat biopsy. *European Urology*.

[45] Hessels D., Klein Gunnewiek J. M. T., van Oort I. (2003). DD3PCA3-based molecular urine analysis for the diagnosis of prostate cancer. *European Urology*.

[46] Luo Y., Gou X., Huang P., Mou C. (2014). The PCA3 test for guiding repeat biopsy of prostate cancer and its cut-off score: a systematic review and meta-analysis. *Asian Journal of Andrology*.

[47] Roobol M. J., Schröder F. H., van Leenders G. L. J. H. (2010). Performance of prostate cancer antigen 3 (PCA3) and prostate-specific antigen in prescreened men: reproducibility and detection characteristics for prostate cancer patients with high PCA3 scores (≥ 100). *European Urology*.

[48] Wei W., Leng J., Shao H., Wang W. (2015). High PCA3 scores in urine correlate with poor-prognosis factors in prostate cancer patients. *International Journal of Clinical and Experimental Medicine*.

[49] Groskopf J., Aubin S. M. J., Deras I. L. (2006). APTIMA PCA3 molecular urine test: development of a method to aid in the diagnosis of prostate cancer. *Clinical Chemistry*.

[50] De Luca S., Passera R., Bollito E. (2014). Comparison of prostate cancer gene 3 score, prostate health index and percentage free prostate-specific antigen for differentiating histological inflammation from prostate cancer and other non-neoplastic alterations of the prostate at initial biopsy. *Anticancer Research*.

[51] Epstein J. I., Walsh P. C., Carmichael M., Brendler C. B. (1994). Pathologic and clinical findings to predict tumor extent of nonpalpable (stage t1 c) prostate cancer. *JAMA*.

[52] Villers A., McNeal J. E., Freiha F. S., Stamey T. A. (1992). Multiple cancers in the prostate. Morphologic features of clinically recognized versus incidental tumors. *Cancer*.

[53] Harnden P., Naylor B., Shelley M. D., Clements H., Coles B., Mason M. D. (2008). The clinical management of patients with a small volume of prostatic cancer on biopsy: what are the risks of progression? A systematic review and meta-analysis. *Cancer: Interdisciplinary International Journal of the American Cancer Society*.

[54] Descotes J.-L. (2019). Diagnosis of prostate cancer. *Asian Journal of Urology*.

[55] Dimakakos A., Armakolas A., Koutsilieris M. (2014). Novel tools for prostate cancer prognosis, diagnosis, and follow-up. *BioMed Research International*.

[56] Kandouci A. B. (2014). Utility of combination of diagnostic tests in early detection of prostate tumors in West Algerian Hospital. *European Journal of Medicine*.

[57] Shimizu T. S., Uchida T., Satoh J., Imai K., Yamanaka H. (1995). Prostate-specific antigen in mass screening for carcinoma of the prostate. *International Journal of Urology*.

[58] Catalona W. J., Richie J. P., Ahmann F. R. (1994). Comparison of digital rectal examination and serum prostate specific antigen in the early detection of prostate cancer: results of a multicenter clinical trial of 6,630 men. *The Journal of Urology*.

[59] Li M., Li X., Guo Y. (2020). Development and assessment of an individualized nomogram to predict colorectal cancer liver metastases. *Quantitative Imaging in Medicine and Surgery*.

[60] Parikh R., Mathai A., Parikh S., Chandra Sekhar G., Thomas R. (2008). Understanding and using sensitivity, specificity and predictive values. *Indian Journal of Ophthalmology*.

